# Effect of Predictive Nursing Combined with Emotional Therapy on Rehabilitation Effect and Psychological State of Patients with Brain Injury after the Operation

**DOI:** 10.1155/2022/4159085

**Published:** 2022-09-27

**Authors:** Xiaying Huang, Haihua Wu

**Affiliations:** ^1^Department of Neurosurgery, Tongde Hospital, Zhejiang Province, China; ^2^Emergency Department, Tongde Hospital, Zhejiang Province, China

## Abstract

Objective. To explore the influence of predictive nursing combined with emotional therapy on the rehabilitation effect and psychological state of patients with brain injury after the operation and to analyze its application value to patients with brain injury after the operation. *Methods*. 70 postoperative patients with brain injury who went to our hospital for diagnosis and treatment were selected as the key figures of this experiment, including 31 female patients and 39 male patients. In order to ensure the uniformity of data, medical staff need to divide patients into an experimental group and a control group through the double-blind method, with 35 cases in each group. The patients in the two groups need to take the relevant diagnosis and surgical treatment measures after admission. The patients in the control group take routine nursing, providing patients with a clean and tidy ward is convenient for patients to manage nursing, and for patients to bring comfortable treatment relief. The patients in the experimental group take predictive nursing combined with emotional therapy, which is to master the basic situation of patients, according to the quality of patients, and develop comprehensive nursing measures for patients. The psychological status, complication incidence rate, treatment effectiveness, and nursing satisfaction of the two groups were compared and analyzed. *Results*. The psychological status, complication incidence rate, nursing efficiency, and nursing satisfaction of patients in the experimental group were significantly better than those in the control group (*P* < 0.05). *Conclusion*. Predictive nursing combined with emotional therapy for patients with brain injury after the operation can effectively alleviate bad mood of patients, reduce the incidence rate of complications, improve the nursing satisfaction of patients, as well as provide patients with high-quality treatment and nursing services. It has a certain clinical application value and is worth popularizing.

## 1. Introduction

Brain trauma is a common disease in neurosurgery. It is mainly caused by the injury of the human brain hit by external objects, resulting in headache, dizziness, confusion, and other phenomena. Brain trauma is easy lead to different clinical complications, such as dizziness, serious cases that will lead to permanent trauma, and greatly reduce the quality of life of patients. This disease has the characteristics of high incidence and high disability rate in the clinic, which has a huge impact on the family and life of patients. Brain trauma is mostly a sudden disease in clinical practice. The injury is serious and the situation is urgent. If there are no active treatment and nursing measures for patients in time, it is easy to lead to patients' forgetting, brain hernia, and other adverse phenomena. Predictive nursing is a comprehensive nursing measure based on medicine, science and life, including diagnosis of a patient's condition, treatment and nursing, prevention, and improvement of treatment effect [1].

Predictive nursing is mainly through the diagnosis of the patient's condition, according to the characteristics of the patient's condition, for patients to make a reasonable treatment plan. Some doctors put forward that predictive nursing has a very high application value in clinical practice, which can understand the patient's condition in all aspects, master the patient's symptoms, and develop a reasonable and effective nursing plan for patients. In clinical practice, predictive nursing can grasp the risk factors of patients in advance, so that patients can take preventive measures timely, reduce the incidence of adverse phenomena, and effectively improve the treatment effect of patients on the premise of ensuring the safety of patients' lives [2]. Affective therapy can improve the therapeutic effect of patients by adjusting their emotional changes. The predictive nursing combined with emotional therapy is to master the basic situation of patients, according to the quality of patients, and develop comprehensive nursing measures for patients.

In order to further improve the rehabilitation effect of patients after traumatic brain injury and improve the survival status of patients, our hospital decided to carry out an analysis of the impact of predictive nursing combined with emotional therapy on the rehabilitation effect and psychological state of patients after traumatic brain injury.

The specific reports are as follows.

## 2. Data and Methods

### 2.1. General Information

A total of 70 patients after TBI who went to our hospital for diagnosis and treatment from March 2021 to March 2022 were selected as the key figures of this experiment, including 31 female patients and 39 male patients. In order to ensure the uniformity of data, medical staff should divide patients into experimental group and control group by double-blind method, with 35 cases in each group. There were 17 female patients and 18 male patients in the experimental group. The average age of patients was (39.3 ± 2.7) years (range, 27–66 years). In the control group, there were 14 female patients and 21 male patients. The average age of patients was (39.41 ± 2.73) years (range, 25–65 years). There was no significant difference in gender, age, and course of disease between these two groups. Our study was approved by the institutional review board of the hospital and was conducted with the ethical principles from the Declaration of Helsinki. Written informed consent was obtained from each participant.

#### 2.1.1. Inclusion Criteria

(1) Patients in the two groups should carry specific data before admission for diagnosis and treatment. (2) Patients after a series of detection and diagnosis of brain trauma diagnostic criteria and patients have taken corresponding surgical treatment nursing measures. (3) Medical staff need to explain the purpose of the experiment to the patient in advance, obtain the consent of the patient, and sign the informed consent with the patient.

#### 2.1.2. Exclusion Criteria

(1) Patients in the process of the study, serious mood fluctuations, refused to cooperate. (2) The patient's body is weak, organ function has an obvious failure, the condition is serious. (3) Patients suffer from cardiovascular diseases or other complications [3].

### 2.2. Methods

Patients in the two groups need to carry out relevant diagnosis and surgical treatment measures after admission. Patients in the control group take routine nursing, while patients in the experimental group take predictive nursing combined with emotional therapy. The *routine* nursing means that medical staff grasp the patient's condition in time, understand the patient's symptoms, and so on. Providing patients with a clean and tidy ward is convenient for patients to manage nursing and for patients to bring comfortable treatment relief. The *predictive* nursing combined with emotional therapy means that excellent and experienced head nurses and nursing staff for a prospective nursing team. The hospital needs regular team members to carry out knowledge and technology training, constantly enhance their nursing skills, and improve their nursing quality.

#### 2.2.1. Routine Nursing

When patients are admitted for diagnosis and treatment, medical staff need to closely observe the value of the patient to the situation, regular examination, detailed record of the patient's examination data, and so on. Most patients have a low understanding of traumatic brain injury and less knowledge. Most of the patient's understanding of the disease is all from the Internet and hearsay, which lack correctness. Even in clinical wrong disease information, is easy to mislead patients. Therefore, medical staff need to timely take knowledge education to patients, through lectures, stories, music, manuals, and other ways to provide patients with an understanding of the disease, help patients master disease knowledge, harm, precautions, and so on, to provide patients with attention. According to the doctor's advice, the patient can be explained how to use the drugs and the dosage and also told to take the drugs on time [4]. Medical and nursing staff need to make regular rounds to patients and greet the treatment of patients, understand the treatment results of patients and so on, and record them in detail. In the process of ward round examination, more than patients communicate, and patients establish a good nurse–patient relationship. In clinical practice, many patients are prone to panic, anxiety, and other psychological phenomena in the face of disease. Bad psychology is easy to lead to more fear of the disease, reduces self-confidence against the disease, affects the treatment of patients, and so on. Medical staff need to closely observe patients' emotional changes, understand patients' bad emotions, and timely communication with patients. In the communication, master the source of patients' bad factors, eliminate patients' bad emotions, and constantly encourage patients. Establish a good nurse–patient relationship with patients in communication and improve patients' self-confidence [5].

#### 2.2.2. Predictive Nursing Combined with Emotional Therapy

Carry out group discussions regularly, each member needs to summarize the outstanding in their work, understand the problem, analyze the problem, and solve the problem. Master the basic situation of patients, according to the quality of patients, and develop comprehensive nursing measures for patients.

1. Respiratory tract foresight nursing: Ventilator therapy is essential for patients with brain trauma in clinical practice. Most patients with traumatic brain injury are in critical condition and often need mechanical ventilation. Health care providers need to improve the treatment of patients while ensuring that they breathe properly. Many bacteria in the human body are carried out through the oral cavity and other ways, so medical staff need to check whether the patient's oral cavity is clean, do a good job of cleaning the teeth and pharynx for patients, and prevent bacteria from carrying out through the oral cavity. Regular daily sputum care for patients, medical staff can gently pat patients on the back. Patients can take sputum care every 2 hours. Patients can be treated with aerosol inhalation every 8 hours. Medical staff need to closely observe the changes in the patient's condition after treatment, and make detailed records and analyses. When performing ventilator-assisted therapy for patients, medical staff need to check whether the ventilator can operate normally, whether oxygen is sufficient, whether there are adverse phenomena, and so on. Before the formal start of ventilator treatment, appropriate masks and other supplies should be selected for patients in advance to ensure that patients can use them normally. Instruct the patient to take the breathing rate and rhythm. The patient was told not to open his mouth as far as possible in the process of treatment to avoid flatulence and other phenomena. In clinical treatment and nursing, if the treatment measures are not appropriate, patients are prone to a series of complications, greatly reducing the treatment effect on patients. In order to effectively prevent the incidence of complications, medical staff need to check all items needed for the treatment of patients in detail, and every cleaning work needs to strictly take aseptic operations to prevent patients from infection and complications caused by bacteria. Medical staff should take active preventive measures for patients and closely observe the changes in patient's condition after treatment and nursing [6].
2. Nutritional support: In clinical practice, most patients with traumatic brain injury are prone to physical fatigue, fainting, confusion, and other phenomena when they are sent to the hospital for treatment. Medical staff need to timely take nutritional support nursing to patients, restore their sanity of patients, and so on. Medical staff can put patients in a good and correct posture to prevent adverse phenomena, such as nutrient fluid reflux when taking nutritional support. Medical staff need to closely observe the patient's treatment and care, and check the patient's pipeline is smooth and clean. To prevent adverse reactions caused by pipe plugs in the process of nutritional support. In the process of treatment, if the patient has nausea, vomiting, and other phenomena, medical staff need to take targeted care of the patient in time, and the condition should be passed through the doctor immediately [7].
3. Drug care: Medical staff need to communicate with doctors when taking drug treatment care for patients, grasp the dose of drug treatment, take time, matters needing attention, and so on. Tell the patient to take the medicine on time, and closely observe the changes in the patient's condition after taking the medicine. Medical staff can know when patients are admitted to take drugs, prevent patients from taking drugs in the wrong way, and reduce the effect of drug treatment and so on. When taking drug treatment for patients, it is necessary to closely check the nature of drugs, infusion speed, vascular elasticity, thickness, etc., and always pay attention to the treatment of patients. When patients take treatment, medical staff need to ensure the normal transportation of patients' drugs and provide high-quality treatment services for patients. Reasonable control of the patient's drug infusion speed, check the transportation situation at all times. If patients need to be transported for a long time, medical staff can choose the thick straight and elastic blood vessels for patients to avoid the adverse reactions that may occur in long-term drug transportation and reduce its harm to the body.
4. Emotional therapy: In clinical practice, medical staff can consciously adjust and change the patients' emotional changes to stimulate the disease. Medical staff can treat patients' diseases by singing, calligraphy, painting, listening to stories, and other measures [8].
5. Other nursing: Medical staff need to closely observe the physical changes of patients, understand the treatment effect of patients, check whether patients have adverse reactions, and so on. Medical staff can help patients develop good living habits, and tell patients after discharge cannot smoke alcohol, overeat, overwork, and so on. Patients can be regularly urged to carry out small exercises to improve ecological immunity [9].

### 2.3. Observation Indicators

Psychological nursing statistics were used for patients, and a Self-Rating Anxiety Scale (SAS) and Self-Rating Depression Scale (SDS) could be issued to patients [10] to record the mood changes of patients at the time of diagnosis and treatment 5 days after treatment in detail. In order to ensure the authenticity of data, medical and nursing staff can guide patients to score but cannot help patients to score by themselves.

1. Each SAS and SDS scale has a total of 20 items, with higher scores indicating more negative emotions.
2. Medical staff need to record in detail the incidence of complications in the treatment process and after treatment of the two groups of patients, pay attention to check whether the patients have headaches, dizziness, confusion and other phenomena, and make detailed records and analysis.
3. Medical staff need to evaluate the treatment efficiency of patients according to their intensive care unit stay time, mechanical ventilation time, hospital stay, etc., to understand the improvement of patient's condition and treatment situation. According to the nursing effect of patients can be divided into four parts namely cure, obvious effect, effective, and ineffective, respectively. A score above 90 is considered as cured, 75–89 is considered as obvious effect, 60–74 is considered as effective, and <60 is considered as ineffective.
4. The nursing satisfaction of the two groups of patients can be statistically analyzed by medical staff through a questionnaire survey. The nursing quality, work performance, and work attitude of medical staff, can be divided into satisfaction, general satisfaction, and satisfaction. A questionnaire survey was carried out on patients with a total of 20 items, with a full score of 100 points. The higher the score, the higher the satisfaction of patients with medical staff.

### 2.4. Statistical Methods

SPSS 25.0 statistical software was used for data analysis. Measurement data were expressed as $\bar{x}\pm s$, *t*-test was used for comparison between groups, count data were expressed as rate and *χ*^2^ test was used. *P* < 0.05 was considered as statistically significant.

## 3. Results

### 3.1. Comparison of Psychological Status Scores between the Two Groups

The SAS and SDS in the experimental group was 55.23 ± 7.41 and 62.39 ± 6.24, respectively, which is significantly higher than that in the control group 54.22 ± 7.71 and 58.80 ± 4.55, respectively. After treatment for 5 days, the SAS in the experimental group was 43.32 ± 4.19, which is lower that that in the control group,48.76 ± 4.34. The SDS in the experimental group was 42.73 ± 4.73, which is significantly lower than that in the control group (see Table 1 for details).

### 3.2. Comparison of Incidence of Complications between the Two Groups

The incidence of complications was 8.57% in the experimental group and 20% in the control group. The incidence of complications in the experimental group was significantly lower than that in the control group (*P* < 0.05). See Table 2 for details.

### 3.3. Comparison of Nursing Efficiency between the Two Groups

The nursing efficiency of the control group was 68.85% and that of the experimental group was 91.42%. The nursing satisfaction of the experimental group was significantly higher than that of the control group (*P* < 0.05). See Table 3 for details.

### 3.4. Comparison of Nursing Satisfaction between the Two Groups

The nursing satisfaction of patients in the control group was 80.00% and the nursing effective rate of patients in the experimental group was 94.28%. The nursing satisfaction of the experimental group was significantly higher than that of the control group (*P* < 0.05). See Table 4 for details.

## 4. Discussion

Brain trauma is a common clinical head injury disease, which is mainly because of the external object hit, so the patient's head visible greater loss, easy to lead to headache, dizziness, confusion, and other phenomena [11, 12]. Brain trauma in clinical practice is mostly a sudden disease, the injury is more serious, the situation is urgent, and medical staff need to timely take targeted treatment and nursing measures for patients. Otherwise, it will lead to different degrees of complications in patients, which will greatly affect the difficulty of treatment in patients. If it is serious, it will lead to permanent trauma in patients and greatly reduce the quality of life of patients. Clinically, early, and timely detection of the disease in patients with mild traumatic brain injury can greatly improve the treatment effect of the patients and also the survival of the patients. But for injury is more critical and serious in the patients, if not taking the correct treatment and measures at right time can easily lead to a series of complications or even death.

Psychotherapy is a social interaction that aims to change the cognitive, behavioral, emotional, and physical feelings of the patient and the patient and involves specifically trained specialists (such as clinical psychologists) to eliminate or mitigate symptoms and problem behaviors. It is usually directed at individuals, but it can also be directed at groups. The intervention is based on a specific theoretical model. Typical models include psychoanalytic therapy, environment-centered therapy, and cognitive behavioral therapy (CBT). Psychoanalysis and patient-centered therapy are difficult to scientifically verify because the interviews are not structured and the number of sessions varies from case to case. Moreover, the mental concepts we deal with are not necessarily observable. As a result, there is very little brain scientific (or empirical) research on these two types of psychotherapy. However, psychoanalysis, which is the oldest in history and has greatly influenced subsequent developments in psychiatry and psychology, has produced many important theoretical concepts and there has been a movement to explore the neurobiological mechanisms underlying this concept. CBT, on the other hand, is structured interview content, and the standard number of sessions has been determined. In addition, behavior and cognition, considered a problem, are extrinsic, in forms that can be observed objectively and can also be assessed quantitatively. Because of this nature, CBT easily follows scientifically validated designs and is currently the best-understood psychotherapy in brain science. Validation of the neurobiological mechanisms of action of CBT is ongoing for various psychiatric disorders, but relatively more reports are for obsessive-compulsive disorder (OCD), phobia, and depression. A disorder characterized by an intense fear of a specific object and avoidance behavior is called a phobia. Objects of fear include blood and heights. When the object of fear is interpersonal interaction, it is known as social anxiety disorder, and in the case of physical symptoms, it is panic disorder. In CBT, this spectrum of phobias, after implementation, significantly reduced activity in the high-limbic regions (tonsil, hippocampus, and parahippocampal), dorsal anterior cingulate cortex (ACC), insula, etc., before treatment, was reported to be at the same level of activity as in healthy individuals. Previous basic research has shown that the amygdala, hippocampus, and olfactory neocortex plays an important role in eliminating fear conditions. CBT for phobia spectrum disorders, considering the elimination of fear-conditioned memories by exposure methods, decreased activity in limbic regions, such as the amygdala and hippocampus after CBT may be closely related to the elimination of learning mechanism. In addition, the island is said to be responsible for the integration of cognition, emotion, and behavior and to be involved in various mental functions, but is specifically noted to play an important role in subjective experiences, especially the internal sensory changes (increased heart rate and pain) caused by the presence of stimuli. On the other hand, back-to-back ACC plays an important role in consciously assessing threatening stimuli and making efforts to control emotional states. Thus, the normalization of brain activity levels in these regions may be associated with the elimination of fear-conditioned memories, the alleviation of overestimation of feared objects and one's physical sensations, and the disappearance of strong emotional responses. In CBT for depression, significant activity changes were found in the ventroexternal prefrontal cortex (VLPFC), limbic regions, such as hippocampus and parahippocampal, posterior cingulate cortex (PCC), and dorsal ACC after treatment. However, the brain regions that changed direction and changed after treatment varied across the studies, and no findings consistent with OCD and phobia spectrum disorders were obtained. There are many subtypes of depression, and its pathological nature is thought to be due to great diversity in severity and the presence or absence of coexisting disorders. VLPFC activity was significantly reduced after remission of depressive symptoms, regardless of whether treatment was medication or CBT. However, in CBT, unlike medication, the dorsal ACC and PCC, and even the amygdala and hippocampus have also shown that it has the potential to ameliorate depressive symptoms by causing some changes. In particular, there is a little activation of the amygdala and hippocampus in depressed patients before treatment even when they show emotional stimulation, but it has also been shown that both become active after treatment. In addition, patients with relatively high amygdala activity during the processing of emotional stimuli also reported greater improvement in depressive symptoms after CBT. From these findings, the limbic region centered in the amygdala did not reach the expected extent in depressed patients, and CBT directed improvement in depressive symptoms by activating its function. In any case, the neural mechanism of action, subtype, and severity of CBT in depression, and considering complications, more elaborate studies are warranted.

The clinical treatment of patients with brain trauma usually requires indwelling a variety of pipelines to improve the physical needs of patients. Medical staff need to make a reasonable treatment plan for patients according to their condition and symptoms. Predictive nursing is a new comprehensive nursing model, which includes diagnosis of a patient's condition, treatment and nursing, prevention to improve the treatment effect, and so on. This nursing model can reduce the risk of infection and improve the rehabilitation effect of patients with traumatic brain injury. In clinical practice, because the condition of patients with traumatic brain injury is more urgent and the speed of change is fast, medical staff need to change traditional passive nursing into active nursing, to improve the quality of nursing services for patients. Medical and nursing staff need to improve patient's condition and treatment effect while ensuring their respiratory tract is clean and their body energy is sufficient [13].

The mental state is one of the basic forms of mental activity, referred to the complete characteristics of mental activity in a certain period, such as attention, fatigue, tension, relief, sadness, and joy. It has both the characteristics of psychological process and individual psychological characteristics, both temporary and stable. It is the intermediary link between psychological process and personality psychological characteristics and constitutes the background of all psychological activities. An individual psychological state is in certain situations, a variety of psychological activity of composite performance, any kind of mental state both the composition of various psychological process and the color of individual differences, also includes many complex psychological processes, not only is a simple split of the psychological process but by the psychological process of compounds with new characteristics. Although the status and function of these components are different in different mental states, mental states are always the comprehensive reflection of mental activities.

The implementation and application of predictive nursing can improve the initiative of patients, meet the treatment needs of patients, and improve the treatment effect of patients on the premise of ensuring the safety of patients' lives. Affective therapy can improve the therapeutic effect of patients by adjusting their emotional changes. Medical staff need to closely observe the emotional changes of patients, can listen to music, singing, calligraphy, and other measures to improve the treatment of patients, improve the effectiveness of patient management, and so on. Predictive nursing combined with emotional therapy has many advantages in clinical application, which are mainly: (a) when patients are confused about the disease, medical staff can timely communicate with patients, relieve patients' bad emotions, and effectively deal with and improve patients' emotions; (b) in the process of treatment, closely observe the treatment of patients, actively take sputum nursing and so on, effectively prevent infection, and reduce the incidence of complications. Medication should be taken according to the doctor's advice, and the medication-taking methods and precautions should be explained to patients to improve the treatment effect of patients [14]. This study mainly adopted predictive nursing combined with emotional therapy for patients in the experimental group. According to the results of this experiment, the psychological status, incidence of complications, nursing efficiency, and nursing satisfaction of patients in the experimental group were better than those in the control group (*P* < 0.05).

## 5. Conclusion

The use of predictive nursing combined with emotional therapy for patients after traumatic brain injury can effectively relieve patients' bad emotions, reduce the incidence of complications, improve patients' nursing efficiency, and nursing satisfaction, and also provide patients with high-quality treatment and nursing services, which has a certain clinical application value and is worth promoting.

## Figures and Tables

**Table 1:** Comparison of psychological status scores between the two groups ($\bar{x}\pm s$).

Constituencies	Number of examples	First hospitalization		Treatment after 5 days	
		SAS	SDS	SAS	SDS
Experimental group	35	55.23 ± 7.41	62.39 ± 6.24	43.32 ± 4.19	42.73 ± 4.73
Control group	35	54.22 ± 7.71	58.80 ± 4.55	48.76 ± 4.34	53.30 ± 5.24
*t*-Value	—	0.251	0.452	6.859	5.580
*P*-value	—	<0.05^∗^	<0.05^∗^	<0.05^∗^	<0.05^∗^

∗p<0.05.

**Table 2:** Comparison of incidence of complications between the two groups ($\bar{x}\pm s$).

Constituencies	Number of examples	Headache	Dizzy	Confusion	Morbidity
Experimental group	35	1	1	1	8.57%
Control group	35	2	2	3	20%
*P*-value	—	—	—	—	<0.05^∗^

∗p<0.05.

**Table 3:** Comparison of nursing efficiency between the two groups (*N*/%).

Constituencies	Number of examples	Heal	Effective	Effective	Void	Efficient
Control group	35	7	5	11	11	24 (68.85%)
Experimental group	35	14	10	8	3	32 (91.42%)
*P*-value	—		—	—	—	0.037^∗^

∗p<0.05.

**Table 4:** Comparison of nursing satisfaction between the two groups (*N*/%).

Constituencies	Number of examples	Satisfied	Generally satisfied	Dissatisfied	Satisfaction with care
Experimental group	35	24	9	2	94.28%
Control group	35	13	15	7	80%
*P*-value	—	—	—	—	<0.05^∗^

∗p<0.05.

## Data Availability

Data supporting this research article are available from the corresponding author or first author on reasonable request.
